# *AKNA* Is a Potential Prognostic Biomarker in Gastric Cancer and Function as a Tumor Suppressor by Modulating EMT-Related Pathways

**DOI:** 10.1155/2020/6726759

**Published:** 2020-05-13

**Authors:** Gang Wang, Dan Sun, Wenhui Li, Yan Xin

**Affiliations:** Laboratory of Gastrointestinal Onco-Pathology, Cancer Institute, The First Affiliated Hospital of China Medical University, Shenyang 110001, Liaoning Province, China

## Abstract

The AT-hook transcription factor, AKNA, is a nuclear protein that affects a few physiological and pathological processes including cancer. Here, we investigated the role of *AKNA* in gastric cancer (GC). By using quantitative real-time polymerase chain reaction (qRT-PCR) and Western blot assays, *AKNA* was found deregulated in both GC cell lines and 32 paired GC tissues. Subsequently, Kaplan-Meier analysis and clinicopathological analysis were conducted using both 32 GC cases' data above and RNA-Seq data of *AKNA* in 354 GC patients and the corresponding clinical-pathological data obtained from The Cancer Genome Atlas (TCGA), and *AKNA* expression was found closely related to location, metastasis, and TNM staging of GC. Then, the potential molecular mechanisms of *AKNA* in GC were explored by gene set enrichment analysis (GSEA), qRT-PCR, and Western blot assays. *AKNA* was found to be a hub gene related to homotypic cell to cell adhesion, regulation of cell to cell adhesion, leukocyte cell to cell adhesion, and regulation of T cell proliferation in GC. GO analysis revealed that *AKNA* involved in the regulation of epithelial-mesenchymal transition (EMT)-related pathways including chemokine signaling pathway, cytokine to cytokine receptor interaction, cell adhesion molecules, and jak-stat signaling pathway in GC. To explore the regulation of *AKNA* expression, *Targetscan* and *TargetMiner* were used to predict the possible miRNA which targeted *AKNA* and found the expression of *AKNA* was negatively correlated to miR-762 which could be sponged by circTRNC18. In conclusion, *AKNA* could function as a tumor suppressor by modulating EMT-related pathways in GC. The expression of *AKNA* might be regulated by circTRNC18/miR-762 axis. *AKNA* could serve as a potential biomarker and an effective target for GC diagnosis and therapy.

## 1. Introduction

Gastric cancer (GC) is the fifth most frequent malignancies and the third most frequent cause of cancer-related death all over the world [1]. Despite great advances in the field of diagnosis and systemic treatment in recent years, the prognosis is unpleasant for GC patients, as the rapid progression to advanced stages and the peculiarity of highly metastatic for GC [2, 3]. In the process of tumor distant metastasis, epithelial-mesenchymal transition (EMT) is a vital and initial molecular step [4]. Therefore, an improved understanding on the underlying mechanisms of the EMT involved in the process of GC metastasis is urgently needed for elucidating the development of relevant therapeutic approaches.

AKNA, also known as the AT-hook transcription factor, is a nuclear protein with AT-hook motif. Increasing evidences indicated crucial function of *AKNA* might exert in multiple cancers. In cervical cancer, single-nucleotide polymorphisms (SNPs) make *AKNA* a susceptibility genetic factor [5]. AKNA directly binds the A/T-rich promoters regions of CD40 and CD40 ligand (CD40L) and coordinately regulates their expression, thereby activate antitumor immune response, while HPV E6, a cervical cancer-related oncoprotein, could downregulate *AKNA* and lead to the progression of cancer [6, 7]. Moreover, by using weighted gene coexpression network analysis (WGCNA), *AKNA* was found to be a hub gene of head and neck squamous cell carcinoma (HNSCC) which is related to the immune response [8]. Recently, Camargo et al. reported that AKNA could regulate EMT in neurogenesis [9]. As is well known that the expression of a certain mRNA could be regulated by circRNA which competitively sponge corresponding miRNA, circRNAs are a unique category of RNA molecules that were first identified in plant viruses in the 1970s [10]. Recently, they have aroused extensive attention as various circRNAs were found to play different roles in multiple diseases, especially in cancers [11, 12]. Growing evidences demonstrate that circRNAs usually regulate tumor progression and metastasis by affecting EMT [13]. CircTRNC18, a circRNA alias hsa_circ_0006772, which is transcripted from *TNRC18* gene, was reported to negatively regulate trophoblast cell migration and EMT via regulating miR-762/Grhl2 axis in preeclampsia [14]. By using bioinformatics tools, we predicted that circTRNC18 could serve as a ceRNA of *AKNA* by competing sponge miR-762. However, the expression and regulatory role of circTRNC18/miR-762/*AKNA* axis in GC progression is not yet clear.

The present study was novel in demonstrating that *AKNA*, a potential target of miR-762, was deregulated in GC and was closely related to location, metastasis, and TNM staging of GC. GSEA analysis revealed *AKNA* could function as a hub gene of GC by regulating EMT-related pathways. *AKNA* might be regulated by circTRNC18/miR-762 axis in GC. The present study provides a promising biomarker and a potential target for GC treatment.

## 2. Materials and Methods

### 2.1. Clinical Specimen Collection

There were 32 fresh primary GC and matched normal gastric epithelial tissues acquired from patients with GC undergoing resection in the First Affiliated Hospital of China Medical University. The samples were immediately collected and placed into RNase-free Eppendorf tubes after resection and put into liquid nitrogen for 5 min, then were put in storage at -80°C for further use. All primary tumor cases and matching normal tissues were verified by qualified pathologists. Permission was obtained from the ethics committee of the First Affiliated Hospital of China Medical University, and informed consent was obtained from patients.

### 2.2. Cell Culture

Five GC cell lines AGS, SGC-7901, BGC-823, MNK-45, HGC-27, and human immortalized normal gastric epithelial cells GES-1 were provided by Genechem Co., Ltd (Shanghai, China). All the cells were maintained and generated in RPMI 1640 (Gibco, USA) supplemented with 10% fetal bovine serum (Hyclone, USA) and cultured at 37°C in 5% CO_2_ atmosphere. Cells were collected when they reached the platform stage.

### 2.3. RNA Extraction and Real-Time PCR

RNA was extracted from GC cells and tissues using miRcute miRNA Kits (Tiangen Biotech Co., Ltd, Beijing, China) following the instructions. Then, 30 *μ*l diethylpyrocarbonate (DEPC)-treated water was used to dissolve the extracted total RNA. The concentration and quality of RNA were determined using a NanoDrop spectrophotometer (Thermo Scientific, USA). Then, extracted RNA underwent reverse transcription using PrimeScript Master Mix (TaKaRa, Japan) for cDNA according to the manual instructions. The primers were constructed and synthesized by Sangon Biotech (Shanghai, China). The qRT-PCR assay was performed, and the expression levels were calculated using the 2 − △△Ct method. Sanger sequencing on the circTRNC18 qRT-PCR product was conducted by Sangon Biotech (Shanghai, China) to validate the specificity of the divergent primers and to confirm the back-splice junction sequence of circTRNC18 was consistent with that from *circBase* database. Glyceraldehyde-3-phosphate dehydrogenase (GAPDH) was used as the internal reference for circTRNC18 and *AKNA* expression detection, and U6 snRNA was used as the internal reference for miR-762 expression detection. The reaction settings of the two-step PCR were as follows: 95°C for 30 s; 40 cycles of 95°C for 5 s, annealing at 55°C for 30 s; dissolving curve at 95°C for 15 s, 60°C for 30 s, and 95°C for 15 s. The primers were as follows: circTRNC18: forward: 5′-GGTGGCAGGGCTTGGAACGG-3′ and reverse: 5′-GCCTTGTCTTGGAGCAGAGCTTC-3′; miR-762: forward: GGGGCTGGGGCCGGGGC and reverse: universal downstream primer; *AKNA*: forward: 5′-GCACCAAGTCCGCAGCATCC-3′ and reverse: 5′-CGCCATCCAGGTCTCCTCCA G-3′; GAPDH: forward: 5′-GAGTCAACGGATTTGGTCGT-3′ and reverse: 5′-TTGATTTTGGAGGGATCTCG-3′; U6: forward: 5′-GGAACGATACAGAGAAGATTAGC-3′ and reverse: 5′-TGGAACGCTTCACGAATTTGCG-3′.

### 2.4. Western Blot

Lysis buffer (Beyotime, China) was used to lyse GC tissues. The harvested protein concentration was quantified by microplate reader using a BCA protein kit (Beyotime, China). The proteins successively underwent electrophoresis, transferred membrane, blocked, and then incubated with primary antibody overnight using anti-AKNA (1 : 500, Proteintech, USA), anti-E-cadherin (1 : 1000, CST, USA), anti-N-cadherin (1 : 1000, CST, USA), anti-vimentin (1 : 1000, CST, USA), and GAPDH (1 : 1000, Origene Co., Ltd., Beijing, China). After incubating with antimouse secondary antibody (1 : 10000, Origene Co., Ltd., Beijing, China), the blot analysis was conducted by an enhanced chemiluminescence system.

### 2.5. Bioinformatics Analysis

RNA-Seq data of *AKNA* in 354 GC patients and the corresponding clinical-pathological data were obtained from TCGA (https://cancergenome.nih.gov/) [15]. The survival curve was plotted using the Human Protein Atlas [16]. The potential molecular mechanisms of *AKNA* in GC were explored by GSEA [17, 18], RNA-seq data of 354 GC patients in TCGA, and collection of annotated gene sets from molecular signatures database v7.0 were used to categorize enriched genes of *AKNA*-low expression group. *Targetscan* and *TargetMiner* were used to predict the possible miRNA which targeted *AKNA* [19, 20].

### 2.6. Statistical Analysis

All statistical analyses were conducted using SPSS25.0 (IBM, NY, USA). Data were presented as mean ± standard error of the mean. The *χ*2 test, Student *t* test, and one-way analysis of variance were used for comparisons. A *P* value less than 0.05 was considered statistically significant.

## 3. Results

### 3.1. Expression of AKNA Was Diminished in GC

qRT-PCR was performed to examine the expression of *AKNA* in GC cell lines and 32 paired GC tissues. The results showed that the expression of *AKNA* was significantly deregulated in GC cells compared to GES-1 (Figure 1(a)). In GC tissues, the expression of *AKNA* was substantially lower than that in paired adjacent noncancerous tissues (Figure 1(b), *P* < 0.05). Furthermore, we conducted western blot to examine the expression of AKNA in 32 corresponding paired GC tissues in protein level, and a consistent expression was observed (Figure 1(c)).

### 3.2. The Expression Patterns of *AKNA* Were Related to the Prognosis of GC Patients and Metastasis of GC

Next, we valued the prognostic role of *AKNA* in GC. By conducting Kaplan-Meier analysis, we found that GC patients with low AKNA expression usually had a worse survival time (5-year survival: low-32% vs high 37%, *P* = 0.012) (Figure 1(d)). To further study the relationship between *AKNA* expression and clinicopathological characters, clinicopathological analysis of 354 GC cases from TCGA database and 32 GC cases from our study were performed, respectively. Results showed that *AKNA* expression in GC was closely related to location, metastasis, and TNM staging (Tables 1 and 2, *P* < 0.05). To further explore the possible mechanism, based on the qRT-PCR result, we detected the expression of several EMT-related markers in AGS and BGC-823 cell lines by using the Western blot assay as BGC-823 cell had a relatively higher expression of *AKNA* than that in AGS. BGC-823 revealed a lower expression of N-cadherin and vimentin and a higher expression of E-cadherin than AGS (Figure 1(e)), which indicated that AKNA might inhibit metastasis by suppressing EMT. Consistent with results above, low expression of *AKNA* had a significantly worse prognosis than that of high *AKNA* expression in GC cases from the TCGA database. All these results demonstrated that the expression of *AKNA* was related to the GC patients' survival and might involve in the regulation of GC metastasis.

### 3.3. AKNA Involved in Regulation of Cell Adhesion and EMT-Related Pathways in GC

To further determine potential functions of *AKNA* in GC progression, based on RNA-Seq data from TCGA, patients were divided into *AKNA*-high and *AKNA*-low groups. The association between *AKNA* expression and related genes signatures were analyzed by GSEA. The genes signatures of homotypic cell to cell adhesion, regulation of cell to cell adhesion, leukocyte cell to cell adhesion, and regulation of T cell proliferation were all highly enriched in patients with *AKNA* high expression, suggesting *AKNA* was involved in these biological processes (Figure 2). KEGG pathway analysis of *AKNA* via GSEA revealed that *AKNA* mainly involved in chemokine signaling pathway, cytokine to cytokine receptor interaction, cell adhesion molecules, and jak-stat signaling pathway, which were closely related to EMT (Figure 3).

### 3.4. miR-762 Was Upregulated in GC and Might Target AKNA

*TargetScan* and *TargetMiner* software were used to predict the possible miRNA which could target *AKNA*. Then, miR-762 was chosen as it has a relatively high score on binding sites prediction with *AKNA* (Figures 4(a) and 4(b)). The expression and function of miR-762 in GC were not completely clear. Firstly, the expression level of miR-762 was assessed by qRT-PCR. Results showed that the expression of miR-762 was upregulated both in GC cells and tissues (Figures 4(c) and 4(d)). Then, the correlation coefficient was calculated, and a medium negative correlation between the expression of miR-762 and *AKNA* was observed in GC (*r* = –0.555, *P* = 0.001; Figure 4(g)), which indicated that miR-762 might target *AKNA*.

### 3.5. circTRNC18 Was Deregulated in GC and Was Negatively Correlated to miR-762

CircRNAs customarily function as miRNA sponges to bind functional miRNAs. As miR-762 has been validated to be sponged by circTRNC18 by a dual-luciferase system in preeclampsia [14], circTRNC18 was chosen for further research. The qRT-PCR assay was conducted to examine the expression of circTRNC18 in GC cells and tissues. The results showed a deregulated expression of circTRNC18 in GC (Figures 4(c) and 4(e)). The correlation analysis revealed a medium negative correlation between the expression of miR-762 and circTRNC18 in GC tissues (*r* = –0.431, *P* = 0.014; Figure 4(f)). These data suggested that circTRNC18 might act as a tumor suppressor and circTRNC18 could serve as a molecular sponge for miR-762 in GC.

## 4. Discussion

Previous studies have revealed the crucial functions of *AKNA* in multiple physiological and pathological processes such as development, immune function, inflammation, and cancer [5, 21, 22]. However, the role of *AKNA* in GC is not yet clear. In this study, by using qRT-PCR and bioinformatics analysis, we found *AKNA* could be a promising biomarker of GC. Firstly, by using qRT-PCR and Western blot, we found *AKNA* was decreased in GC tissues in mRNA and protein levels, respectively. Manzo et al. conducted histology and immunohistochemistry (IHC) to evaluate the expression of AKNA in cervical biopsies of 12 cases of hysterectomy, which contains normal epithelium, cervicitis, and infiltrating squamous cell carcinoma (SCC), and found a substantial decrease of AKNA production in dysplasia area and SCC compared to normal cervical epithelium [7]. Our results were consistent with this trend.

Since the sample size of 32 is limited to conduct further analysis, the prognostic value of *AKNA* was also evaluated through a dataset which contains 354 GC cases obtained from the TCGA database. A significant correlation between *AKNA* low expression and poor OS was found in GC. More interesting thing is that the expression level of *AKNA* was correlated with tumor location, metastasis, and TNM staging. It could be inferred that *AKNA* could be a prognostic biomarker for GC.

In addition, our GSEA result revealed that *AKNA* could regulate GC progression via various pathways like chemokine signaling pathway, cytokine to cytokine receptor interaction, cell adhesion molecules, and Janus kinase/signal transducer and activator of transcription (jak-stat) signaling pathway. Chemokines are a class of cytokines that act as signaling molecules, regulating immune and inflammatory responses. In the tumor microenvironment, chemokines were released to regulate cellular migration and cell-cell interactions, thereby mediate the balance between responses of antitumor and protumor. What is more, chemokines are also involved in other tumor progression processes such as tumor cell growth, angiogenesis, and tumor metastasis [23]. It is well known that jak-stat signaling is activated in multiple tumors including GC and implicated in tumor formation and metastatic progression, and cytokine IL-6 is a major activator of jak2/stat3 signaling [24]. Liu et al. reported that GH and inflammatory cytokines (TNF-*α*, IL-1*β*, and IL-6) expression were significantly downregulated after *AKNA* silencing [25]. Our results indicated that when the expression of *AKNA* was dysregulated, the balance between responses of antitumor and protumor would be broken as a result of the abnormal activation of the chemokine signaling pathway and the jak-stat signaling pathway.

Moreover, we found that dysregulated *AKNA* was related to cell to cell adhesion molecules in GO analysis. It is well known that the most important features of a malignant tumor are invasion and metastasis, and EMT is the initial step for tumor invasion and metastasis. The EMT is a process during which epithelial cells are gradually shifted into mesenchymal cells, which promotes the metastasis of tumor cells. During EMT, differentiated epithelial cells lose their apical-basal polarity and epithelial adhesion and acquire a myofibroblastic phenotype, with the change of multiple EMT-markers such as E-cadherin, N-cadherin, vimentin, and *α*-smooth muscle actin, which is accompanied by enhanced cell migration and invasion capabilities. Camargo et al. reported that knocking down of *AKNA* in normal murine mammary gland epithelial cells during an EMT process induced by TGF*β*1 led to ZO-1 tight junction protein and attenuated the rearrangement of actin fibres from the junctions to stress fibres, which indicated that the important role of *AKNA* in the regulation of cell adhesion in EMT [9]. Our Western blot assay result on EMT markers detection in AGS and BGC-823 cells was in line with this. It has been reported that in HNSCC, through WGCNA, *AKNA* was found to function as a hub gene that might involve in immune response, inflammatory response, and formation of the tumor microenvironment [8]. Our GSEA results revealed that the same effect of *AKNA* might also exist in GC. What is more, we found that dysregulated *AKNA* is probably related to distant metastasis of GC, and dysregulated *AKNA* could lead to an attenuated cell adhesion via inducing EMT in GC. Considering that AKNA involves in signaling pathways related to the genesis and progression of GC, *AKNA* could be a promising new therapeutic target for GC. However, as this conclusion is mainly drawn based on bioinformatic analysis, further experiments, including both in vitro and in vivo, are needed to explicit the potential role of *AKNA* in GC.

Finally, we explored the molecular mechanism underlying the regulation of *AKNA* in GC. Through using bioinformatic tools, we predicted the potential targets of *AKNA* and chose the circTRNC18/miR-762 axis for the further research. In recent years, increasing studies have reported the remarkable role of noncoding RNAs (ncRNAs) in tumorigenesis and progression [26]. CircRNAs, a new class of ncRNAs, which are formed via back-splicing and have neither 5′–3′ polarities nor polyadenylated tails structural, have gradually gained attention [27]. Increasing convincing evidences demonstrated that a large amount of circRNAs were dysregulated in multiple cancers including GC and could serve as sponges for miRNAs to regulate the expression of downstream targets. Du et al. reported that circ-PRMT5 was significantly upregulated in GC and could serve as miR-145 and miR-1304 “sponge,” thereby upregulating expression of *myc*, an oncogene, and promoting GC progression [28]. Dai et al. found that circGRAMD1B was downregulated in GC and confirmed that circGRAMD1B could serve as a tumor suppressor in GC by sponging miR-130a-3p via *in vivo* and *in vitro* experiments [29]. It was reported that circTRNC18 is negatively regulated trophoblast cell migration and EMT via regulating miR-762/Grhl2 axis in preeclampsia [14]; however, the role of circTRNC18 in GC is still unclear. Therefore, we firstly detected circTRNC18 in GC cells and tissues and demonstrated that circTRNC18 was decreased in GC. Moreover, we found miR-762 was upregulated in GC and negatively related to the expression of circTRNC18, which was consistent with the dual-luciferase reporter results of binding validation between circTRNC18 and miR-762 in the previous study [14], indicating that circTRNC18 might be a tumor suppressor in GC by sponging miR-762. By using bioinformatic tools and correlation analysis, we indicated that *AKNA* might be the target of miR-762 in GC; however, there is further need for a dual-luciferase reporter assay to confirm their direct binding.

## 5. Conclusion

Taken together, *AKNA* is downregulated in GC. *AKNA* is a potential tumor suppressor, and it might function in GC through affecting EMT-related pathways including chemokine signaling pathway, cytokine to cytokine receptor interaction, cell adhesion molecules, and jak-stat signaling pathway. *AKNA* might be regulated by circTRNC18/miR-762 axis. *AKNA* could serve as a potential biomarker and an effective target for GC diagnosis and therapy.

## Figures and Tables

**Figure 1:** The expression pattern of *AKNA* in human GC. (a) The expression of *AKNA* in GC cell lines and GES-1 was detected by qRT-PCR. (b) *AKNA* expression in 32 GC and paired normal tissues was detected by qRT-PCR. Data are means ± SEM. ∗*P* < 0.05. (c) Western blot assay was performed to determine AKNA expression in 32 GC tissues and paired normal tissues. (d) Prognostic value of the expression of *AKNA* in 354 patients with GC in the TCGA database. (e) Western blot assay was performed to determine EMT-related markers expression in AGS and BGC-823 cells.

**Figure 2:** GO analysis of *AKNA* in GC. The association between *AKNA* expression and related gene signatures was analyzed by GSEA followed by GO analysis.

**Figure 3:** KEGG analysis of *AKNA* in GC. The association between *AKNA* expression and related gene signatures were analyzed by GSEA followed by KEGG analysis.

**Figure 4:** The correlation of *AKNA* and circTRNC18/miR-762 axis in GC. (a, b) One of the most possible miRNA targeted *AKNA* was predicted by *Targetscan* and *TargetMiner*. *AKNA* had multiple potential binding sites with miR-762. (c) The expression of circTRNC18 and miR-762 in GC cell lines and GES-1 was detected by qRT-PCR. Data are means ± SEM. ∗*P* < 0.05, ∗∗*P* < 0.01. (d) The expression of miR-762 in 32 GC and paired normal tissues was detected by qRT-PCR. Data are means ± SEM. ∗*P* < 0.05. (e) The expression of circTRNC18 in 32 GC and paired normal tissues was detected by qRT-PCR. Data are means ± SEM. ∗*P* < 0.05. (f) Pearson's correlation coefficient was calculated between miR-762 and circTRNC18 expression in GC. *r* = –0.431, *P* = 0.014. (g) Pearson's correlation coefficient was calculated between miR-762 and *AKNA* expression in GC. *r* = –0.555, *P* = 0.001.

**Table 1:** The relationship between *AKNA* expression level and clinicopathological factors in 354 GC cases from the TCGA database.

Characteristics	*N*	Expression of *AKNA*		*χ*2	*P*
		Low	High		
Gender	354	101	253	0.108	0.742
Male	229	64 (27.9%)	165		
Female	125	37 (29.6%)	88		
Age(years)	351	101	250	3.41	0.065
≤65	150	37 (24.7%)	113		
>65	201	64 (31.8%)	137		
Tumor sites	340	96	244	13.256	0.004
Gastroesophageal junction	39	16 (41.0%)	23		
Cardiac	45	19 (42.2%)	26		
Fundus/body	124	23 (18.5%)	101		
Antrum	132	38 (28.8%)	94		
WHO's histological types	103	24	79	3.005	0.391
Tubular Ade.					
Moderately Diff.	5	2 (40.0%)	3		
Poorly Diff.	68	18 (26.5%)	50		
Mucinous Ade.	11	1 (9.1%)	10		
Signet ring cell car.	19	3 (15.8%)	16		
Lauren's types^a^	233	65	168	1.668	0.196
Intestinal type	161	49 (30.4%)	112		
Diffuse type	72	16 (22.2%)	56		
Depth of invasion	354	101	253	2.339	0.505
T1	18	7 (38.9%)	11		
T2	62	20 (32.3%)	42		
T3	12	2 (16.7%)	10		
T4	262	72 (27.5%)	190		
Ln metastasis	318	83	235	2.375	0.498
N0	89	25 (28.1%)	64		
N1	66	19 (28.8%)	47		
N2	73	14 (19.2%)	59		
N3	90	25 (27.8%)	65		
Distant metastasis	338	97	241	9.337	0.002
M0	315	84 (26.7%)	231		
M1	23	13 (56.5%)	10		
TNM staging	306	82	224	15.012	0.002
I	42	15 (35.7%)	27		
II	57	15 (26.3%)	42		
III	184	39 (21.2)	145		
IV	23	13 (56.5%)	10		

Ade.: adenocarcinoma; Diff.: differentiated; Car.: carcinoma; Ln.: lymph node.^a^Lauren's types data of 121 GC cases is unavailable.

**Table 2:** The relationship between AKNA expression level and clinicopathological factors in 32 GC cases.

Characteristics	*N* = 32	Expression of *AKNA*		*χ*2	*P*
		Low (*N* = 16)	High (*N* = 16)		
Gender					0.685∗
Male	24	13 (54.2%)	11		
Female	8	3 (37.5%)	5		
Age(years)				4.800	0.028
≤60	12	9 (75.0%)	3		
>60	20	7 (35.0%)	13		
Borrmann's types					0.433^∗^
I+II	9	6 (66.7%)	3		
III	23	10 (43.5%)	13		
Lauren's types				0.533	0.465
Intestinal type	12	7 (58.3%)	5		
Diffuse type	20	9 (45.0%)	11		
Depth of invasion				3.463	0.063
T1~T3	11	3 (27.3%)	8		
T4	21	13 (61.9%)	8		
Ln metastasis				8.533	0.003
N0	12	2 (16.7%)	10		
N1~N3	20	14 (70.0%)	6		
Distant metastasis					1.000^∗^
M0	31	15 (48.4%)	16		
M1	1	1 (100%)	0		
TNM staging				1.166	0.280
I+II	13	5 (38.5%)	8		
III+IV	19	11 (57.9%)	8		

^∗^Fisher's exact test. Ln.: lymph node.

## Data Availability

The data used to support the findings of this study are available from the corresponding author upon request.
